# lncRNA MALAT1 Promotes Diabetic Nephropathy Progression via miR-15b-5p/TLR4 Signaling Axis

**DOI:** 10.1155/2022/8098001

**Published:** 2022-07-21

**Authors:** Zijun Yang, Dongxu Song, Yulin Wang, Lin Tang

**Affiliations:** Department of Nephropathy, The First Affiliated Hospital of Zhengzhou University, Zhengzhou, China

## Abstract

**Objective:**

The long noncoding RNA metastasis-associated lung adenocarcinoma transcript 1 (MALAT1) are closely associated with the pathogenesis of diabetic nephropathy (DN). But a complete mechanism for MALAT1 in DN has yet to be identified. This study investigated the effect of MALAT1 on DN through the regulation of miR-15b-5p/TLR4 signaling.

**Method:**

Renal tissues were collected from DN patients. Human renal tubular epithelial cells (HK-2) were used as a model of DN induced by high glucose (HG). We then measured the viability, apoptosis, and inflammatory cytokine levels of HK-2 cells using the corresponding assays. Following transfections of si-MALAT1, si-MALAT1+miR-15b-5p inhibitor, or si-MALAT1+vector TLR4 into HG-stimulated HK-2 cells, cell viability, apoptosis, and inflammatory cytokines were again measured. Furthermore, dual-luciferase reporter assay validated the interactions of MALAT1/miR-15b-5p and miR-15b-5p/TLR4. In addition, the interaction between MALAT1 and miR-15b-5p was investigated by RNA immunoprecipitation (RIP).

**Results:**

A significant upregulation of MALAT1 was observed in DN kidney tissues, as well as in HG-stimulated HK-2 cells. MALAT1 knockdown attenuates the inhibition of cell viability, apoptosis, and inflammatory response induced by HG in HK-2 cells. Moreover, a miR-15b-5p inhibitor or TLR4 overexpression reversed the above effects induced by MALAT1 knockdown.

**Conclusion:**

These results indicate that reduced MALAT1 ameliorates HG-stimulated HK-2 cell damage through an inhibition of the miR-15b-5p/TLR4 axis. MALAT1 may serve as a biomarker and potential therapeutic target for DN.

## 1. Introduction

The leading cause of end-stage renal disease in the world is diabetic nephropathy (DN), a serious microvascular complication of diabetes [1, 2]. With unremitting efforts, the diagnosis and treatment of DN have advanced greatly [3]. However, the progression of DN cannot be prevented owing to its complicated pathological mechanisms, which in turn results in huge economic burdens on many families and society. Therefore, there is an urgent need to explore the pathogenesis of DN for effective therapies.

Recently, emerging evidence has indicated that tubular impairment induced by hyperglycemia is more serious than glomerular lesions. It may be the main cause of early DN [4, 5]. Previous findings have revealed that apoptosis and inflammation are the major pathogenesis mechanisms of DN, playing vital roles in accelerating the progression and deterioration of DN [6]. Long noncoding RNAs (lncRNAs) contain more than 200 nucleotides and contribute to the pathogenesis and physiology of many diseases, such as DN [7]. The lncRNA, metastasis-associated lung adenocarcinoma transcript 1 (MALAT1), was first identified in lung cancer [8]. Recently, evidences indicated that MALAT1 has shown a close relationship with DN [9, 10]. For example, in the study by Zhang et al. [11] and Liu et al. [12], high glucose (HG) induced epithelial-to-mesenchymal transition and pyroptosis mediated by MALAT1 in human renal tubular epithelial cells (HK-2). However, there are still few studies on the effect of MALAT1 in DN tubular epithelial cell apoptosis and inflammation, and more investigations are needed to prove this.

MicroRNAs (miRNAs) are evolutionarily conserved noncoding RNAs encoded by higher eukaryotes' genomes. They regulate cell growth and development by interacting with the mRNA of target genes, which activates the silencing complex (RISC) to degrade or block the mRNA. miRNAs have been shown to contribute to DN pathogenesis [13–15]. Researchers previously discovered that DN patients had decreased levels of microRNA 15b-5p (miR-15b-5p) which suppressed inflammation, inhibited apoptosis, and repressed oxidative stress in HG-induced podocyte lesions [16]. Many evidences have demonstrated that DN [17, 18] bears a high sensitivity to Toll-like receptor 4 (TLR4) that promotes the release of inflammatory cytokines like tumor necrosis factor- (TNF-) *α*, interleukin- (IL-) 6, and IL-1*β* [19, 20]. But whether miR-15b-5p participated in DN tubular epithelial cell damage by regulating TLR4 has not been studied.

lncRNAs regulate various biological processes by preventing miRNA-mediated target-mRNA degradation. As miRNA sponges, they form a well-established lncRNA-miRNA-mRNA competitive regulatory axis. For example, ablation of myocardial infarction-associated transcript (MIAT) mitigated HG-induced inflammation and podocyte apoptosis through the miR-130a-3p/TLR4 pathway [21]. Cyclin-dependent kinase inhibitor 2B antisense RNA 1 (CDKN2B-AS1) negatively regulated miR-424-5p and then targeted high-mobility group AT hook 2 (HMGA2) to promote extracellular matrix aggregation in mesangial cells [22]. Moreover, the bioinformatics analysis indicated that MALAT1 and miR-15b-5p have two complementary sequences, and miR-15b-5p binds to the 3′-untranslated region (3′-UTR) of TLR4.

Thus, we hypothesized that the MALAT1/miR-15b-5p/TLR4 axis might contribute mechanistically to the progression of DN. So far, there is no study on this pathway in the pathogenesis involved in DN. This study was conducive to identifying potential therapeutic targets for DN.

## 2. Material and Methods

### 2.1. Collection of Human Renal Tissues

We collected DN renal tissues (*n* = 18) from DN patients diagnosed by renal biopsy in the Department of Nephrology, the First Affiliated Hospital of Zhengzhou University. The adjacent noncancerous tissues (*n* = 16) from patients who underwent tumor resection for renal carcinoma were selected as controls. These patients did not have diabetes or other kidney diseases. The hospital ethics committee approved the study, and all patients provided informed consent before participating.  Table 1 shows the clinical features of DN patients.

### 2.2. Cell Culture

We purchased HK-2 cells from Procell (Wuhan, China) and cultured them in DMEM (1 g/L glucose) supplemented with 1% penicillin/streptomycin and 10% fetal bovine serum (Gibco, USA) and placed them at 37°C with 5% CO_2_. We treated HK-2 cells with normal glucose (NG) (5.6 mM glucose), hyperosmotic solution (HM) (5.6 mM glucose+24.4 mM mannitol), and high glucose (HG) (30 mM glucose).

### 2.3. Quantitative Real-Time- (qRT-) PCR

We extracted total RNA using TRIzol (Invitrogen, USA) and measured the concentration and purity using the NanoDrop One ultramicroultraviolet spectrophotometer. Then, the extracted RNA was reversely transcribed into cDNA with Thermo Fisher Revert Aid First-Stand cDNA Synthesis Kits (Invitrogen, #K1622, USA) or miRNA First-Strand cDNA Synthesis (tailing reaction) (Shanghai, China, B532451-0020). Finally, qPCR was conducted using a SYBR Green PCR Master Mix kit (Thermo Fisher Scientific, USA). The temperatures were set as follows: predenaturation at 95°C for 2 minutes, denaturation at 95°C for 15 seconds, and annealing/extension at 60°C for 1 minute with a total of 40 cycles. We analyzed the relative gene expression levels using the 2^−*ΔΔ*Ct^ method. *β*-Actin (for lncRNA) and U6 (for miRNA) were used as endogenous controls, respectively. The specific primers were listed in Table 2.

### 2.4. Cell Viability Assay

Prepare the transfected cell suspension and inoculate the cells into 96-well plates, with 2 × 10^3^ cells/100 *μ*L per well, and preincubate in the 37-degree incubator for 24 hours, then add 10 *μ*L CCK-8 solution (Enzyme Biotech, Nanjing, China) to each well, and measure the absorbance value at 450 nm using a microplate reader (Molecular Devices, Sunnyvale, CA, USA) after two hours.

### 2.5. Apoptosis Assay

We use the terminal deoxynucleotidyl transferase dUTP nick-end labeling (TUNEL) BrightRed Apoptosis Detection Kit to detect apoptosis (Enzyme Biotech, Nanjing, China). When apoptosis occurs, intracellular specific endonuclease is activated, chromatin DNA between nucleosomes is specifically cut, and DNA is degraded into 180-200 bp fragments. The 3′-hydroxy (3′-OH) end produced by DNA molecular breakage can bind to tetramethylrhodamine deoxyuridine triphosphate (TMR red dUTP) under the action of terminal deoxyribonucleotide transferase (TdT) The apoptotic nucleus were labeled red, and both the apoptotic and nonapoptotic cells were dyed blue by 4′,6-diamidino-2-phenylindole (DAPI). Apoptotic cells were observed and counted under a fluorescence microscope. The percentage of apoptotic cells was analyzed by Image-Pro Plus 6.0 software (Media Cybernetics, Rockville, MD, USA).

### 2.6. Enzyme-Linked Immunosorbent Assay

Enzyme-linked immunosorbent assay kits (CUSABIO, Wuhan, China) were used to measure the levels of TNF-*α*, IL-1*β*, and IL-6.

### 2.7. Western Blotting

Total proteins were obtained from HK2 cells from all groups (NG, HG, HG+si-MALAT1, HG+si-MALAT1+miR-15b-5p inhibitor, HG+mimics negative control (NC), and HG+miR-15b-5p mimics) using Radioimmunoprecipitation Assay (RIPA) Lysis Buffer on ice, and the concentration was measured by BCA Protein Assay Kit (Solarbio, PC0020). Each protein sample was taken 40 *μ*g. After separation by 10% sodium dodecyl sulfate polyacrylamide gel electrophoresis (SDS-PAGE), the proteins were transferred to polyvinylidene difluoride (PVDF) membranes. The membrane was sealed with 5% skimmed milk at 37°C for 2 h and then was incubated with the primary antibody TLR4 (Abcam, ab22048) overnight at 4°C. *β*-Actin was used as the internal reference to calculate the relative expression of each protein. Tris-Buffered Saline Tween (TBST) washed the membrane for 3 times, each time for 15 min. Finally, the secondary antibody (Abcam, ab13556, anti-mouse) labeled by horseradish peroxidase (HRP) was added and incubated at 37°C for 2 h. After the membrane was washed and colored by ECL, signals were detected using the ChemiDocMP Imaging System (Bio-Rad, Shanghai, China).

### 2.8. Cell Transfection

We seed HK-2 cells into 6-well plates. The si-MALAT1 and miR-15b-5p mimics and their corresponding controls (si-NC, mimics NC) (GenePharma, Shanghai, China) were transfected with Lipofectamine 3000 (Invitrogen, USA). Next, we treated the transfected cells with NG or HG.

### 2.9. Plasmid Construction and Dual-Luciferase Reporter Assay

The potential binding site sequence of wild-type MALAT1 or TLR 3′-UTR was inserted into psiCHECK-2 to construct luciferase reporter gene plasmid named MALAT1-Wt or TLR 3′-UTR-Wt. Similarly, MALAT1-Mt or TLR 3′-UTR-Mt was established using mutated sequences, and then, miR-15b-5p mimics or mimics NC was cotransfected into HK-2 cells, respectively, using Lipofectamine 3000 (Invitrogen, USA). The cells were lysed and various working fluids were added with the dual luciferase reporter assay kit (Promega, China). Finally, the luciferase activity was measured using Luminometer chemiluminescence detector and the data were analyzed.

### 2.10. RNA Immunoprecipitation (RIP) Assay

Using the Magna RIP Kit (Millipore, USA), we examined the interaction between MALAT1 and miR-15b-5p. Anti-Ago2 and control IgG antibodies were used (Millipore, USA). After that, the precipitates were used for cDNA synthesis and qRT-PCR.

### 2.11. Statistical Analysis

We used SPSS 26.0 software for statistical analysis as well as GraphPad Prism 8.0 software for graphing. An independent sample *T* test was used to compare two samples where the variables were normal distributed. Multivariate samples with homogeneous variance were compared via one-way ANOVA, and multiple comparisons were assessed using the LSD test. Multivariate samples with heterogeneous variance were compared with Welch test, and multiple comparisons were done with Dunnett's test. Statistical significance was defined as *p* < 0.05.

## 3. Results

### 3.1. HG Induces MALAT1 Expression

MALAT1 expression was measured using qRT-PCR analysis in DN (*n* = 18) and in normal tissues (*n* = 16). MALAT1 was significantly upregulated in DN tissues compared with normal tissues (Figure 1(a)).

Next, HK-2 cells were treated with NG, HM, or HG for 12, 24, 36, or 48 h to assess how much HG affects MALAT1 expression. Then, MALAT1 levels were examined. Our results showed that MALAT1 expression in HK-2 cells was significantly elevated by HG compared with the NG group (Figure 1(b)). However, MALAT1 expression was almost the same at 36 and 48 h. MALAT1 expression did not change in the HM group, indicating that the HG-stimulated increase of MALAT1 was not caused by osmotic pressure. In addition, miR-15b-5p level was also measured in HK-2 cells under NG, HM, or HG conditions. Compared with the NG or HM group, miR-15b-5p was downregulated more than 2-fold after 36 h of HG stimulation (Figure 1(c)).

### 3.2. Knockdown of MALAT1 Attenuates HK-2 Cell Viability Inhibition, Apoptosis, and Inflammation Induced by HG

MALAT1 was further studied in DN using HG-incubated HK-2 cells which were transfected with si-MALAT1 or their corresponding control small-interfering RNAs under HG condition. The levels of MALAT1 were reduced markedly after transfection with si-MALAT1 (Figure 2(a)). Furthermore, HG treatment decreased cell viability (Figure 2(b)), promoted cell apoptosis (Figures 2(c) and 2(d)), and notably increased the levels of TNF-*α*, IL-1*β*, and IL-6 (Figures 2(e)–2(g)) in HK-2 cells. Importantly, these HG-induced effects in HK-2 cells were alleviated by MALAT1 knockdown compared with the HG group or HG+si-NC group.

### 3.3. MALAT1 Inhibits Cell Viability and Promotes Cell Apoptosis and Inflammation by Targeting miR-15b-5p

As a miRNA sponge, lncRNA is widely known to regulate a wide variety of physiological processes. We performed bioinformatics analyses using TargetScan and PicTar programs to identify two binding sites and two complementary sequences shared by MALAT1 and miR-15b-5p (Figure 3(a)).

To confirm the interaction between MALAT1 and miR-15b-5p, the luciferase reporter plasmids MALAT1-Wt1 and MALAT1-Mt1 or MALAT1-Wt2 and MALAT1-Mt2 were constructed. HK-2 cells were cotransfected with miR-15b-5p mimics or mimics NC. Dual-luciferase reporter analysis demonstrated that miR-15b-5p mimics induced a >50% reduction in luciferase activity in MALAT1-Wt1 transfectants, whereas the activity of MALAT1-Mt1 did not change (Figure 3(b)). Similar results were obtained from MALAT1-Wt2 and MALAT1-Mt2 (Figure 3(c)). Furthermore, the Ago2 RIP showed that MALAT1 and miR-15b-5p were abundant in the same complex, that is, both MALAT1 and miR-15b-5p were pulled down by the Ago2 antibody (Figure 3(d)), further verifying their binding potential. The expression level of miR-15b-5p was detected using qPCR in HK-2 cells transfected with si-MALAT1 under NG and HG conditions. As shown in Figure 3(e), knockdown of MALAT1 under HG condition significantly increased miR-15b-5p levels compared with the si-NC group, and similar results were obtained under NG condition. Next, we evaluated TLR4 levels, cell viability, apoptosis, and TNF-*α* levels after si-MALAT1 and miR-15b-5p inhibitor were transfected into HK-2 cells. TLR4 mRNA and protein levels were downregulated (Figures 3(f) and 3(g)), HK-2 cell viability increased (Figure 3(h)), apoptosis decreased (Figures 3(i) and 3(j)), and TNF-*α* levels were downregulated (Figure 3(k)) after transfection with si-MALAT1 under HG condition. In contrast, the opposite results were obtained after transfecting HK-2 cells with si-MALAT1 and miR-15b-5p inhibitor. These results suggest that MALAT1 targets miR-15b-5p to inhibit cell viability and promote cell apoptosis and inflammation.

### 3.4. miR-15b-5p Negatively Regulates TLR4 and MALAT1 Regulates TLR4 Expression via miR-15b-5p

Currently, increasing studies emphasized the importance of the lncRNA-miRNA-mRNA regulatory network. Bioinformatics tools predicted miR-15b-5p targets TLR4. The target site is shown in Figure 4(a). The binding potential between miR-15b-5p and TLR4 was validated by dual-luciferase reporter gene assay. TLR4 3′-UTR-Wt or TLR4 3′-UTR-Mt plasmid vector and miR-15b-5p mimics or mimics NC were cotransfected into HK-2 cells. The results indicated that miR-15b-5p mimics inhibited the luciferase activity of TLR4 3′-UTR-Wt by almost 50%, while miR-15b-5p mimics had little effect on the activity of TLR4 3′-UTR-Mt (Figure 4(b)). Compared with the HG and HG+mimics NC groups, TLR4 protein expression was significantly reduced in the HG+miR-15b-5p mimics group (Figure 4(c)). To determine whether MALAT1 regulates TLR4 via miR-15b-5p, cell viability, apoptosis, and TNF-*α* levels were measured after si-MALAT1 or si-MALAT1+vector TLR4 transfection of HK-2 cells treated with HG. The results showed that HK-2 cell viability increased (Figure 4(d)), apoptosis decreased (Figures 4(e) and 4(f)), and TNF-*α* levels were downregulated (Figure 4(g)) after transfection with si-MALAT1, whereas TLR4 overexpression reversed the above effects. In summary, our findings indicated that miR-15b-5p negatively regulates TLR4 and MALAT1 enhanced TLR4 expression via miR-15b-5p.

## 4. Discussion

Inflammation may play a crucial role in the pathophysiology of DN, as evidence is mounting [23–25]. Hyperglycemia can stimulate the secretion of inflammatory cytokines, induce apoptosis, and generate numerous reactive oxygen species, resulting in injury to renal tubular epithelial cells [26], renal endothelial cells [27], mesangial cells [28, 29], and podocytes [30].

Recent findings have indicated that lncRNAs and miRNAs play critical roles in DN progression by regulating cellular inflammation [31–33]. Among them, the lncRNA MALAT1 and miR-15b-5p are often implicated in DN. MALAT has been found to be upregulated in DN and recruit methyltransferase G9a to inhibit klotho expression in HG-stimulated glomerular endothelial cell injury [27]. As is similar to previous studies, we observed that the level of MALAT1 increased in DN and downregulation of MALAT1 attenuated HK-2 cell viability inhibition, apoptosis, and inflammation induced by HG.

Previously, the expression of miR-15b-5p in HG-cultured HK-2 cells was reported to decrease markedly and miR-15b-5p ameliorated the apoptosis caused by HG by activating the mTOR pathway and inhibiting JNK signaling [34]. Similarly, Chang et al. demonstrated that miR-15b-5p was downregulated while CDKN2B-AS1 and wingless-type family member 2B (WNT2B) were upregulated in DN serum and HG-incubated human mesangial cells (HMC). CDKN2B-AS1 regulated HMC viability, inflammation, and ECM accumulation through the miR-15b-5p/WNT2B axis [35]. Notably, a recent study revealed that the MALAT1/miR-15b-5p/MAPK1 and mTOR signaling pathways were essential to the development of coronary atherosclerosis [36]. Inspired by this, we investigated the relationship between MALAT1 and miR-15b-5p in HG-induced HK-2 cells. We are the first to show the interaction between them using DN models.

The bioinformatics analysis results of our study suggested that miR-15b-5p could target TLR4. We further performed dual-luciferase reporter gene assay to validate their interplay. Accumulating evidences suggested that TLR4 is upregulated in DN [37] and is highly expressed in HG-stimulated podocytes [30] and HK-2 cells [38]. Liu et al. [39] demonstrated that knockdown of TLR4 attenuated the HG-stimulated podocyte cell apoptosis and reduced cell viability and inflammation. Several miRNAs exert their effects by targeting TLR4. For example, Zhu et al. revealed that miR-195 resulted in inhibition of macrophage proliferation and reduction of the release of inflammatory cytokines via the TLR4/NF-*κ*B axis in DN rats [40]. However, the association between miR-15b-5p and TLR4 in DN has seldom been reported.

Previous findings have indicated that MALAT1 antagonizes miRNA function and triggers the TLR4 pathway by using various disease models. Recently, MALAT1 was shown to increase inflammatory cytokine release by binding with miR-20a and activating TLR4 during periodontal inflammation [41]. Similarly, He et al. showed that human pulmonary artery smooth muscle cells were promoted to proliferate and migrate by MALAT1 through regulating TLR4 expression [42]. However, none of these studies focused on DN. Thus, we hypothesized that MALAT1 may regulate TLR4 through miR-15b-5p in the process of occurrence and development of DN. This hypothesis was verified in subsequent experiments.

However, our study has a few limitations. Firstly, we only detected MALAT1 in renal DN tissues and normal tissues but did not examine miR-15b-5p and analyze the correlation between them. Secondly, there was a need to increase sample size to improve accuracy. Thirdly, the specific regulatory mechanisms of MALAT1 remain to be further studied.

To summarize, we observed that the expression of MALAT1 was significantly higher in renal DN tissues. Knockdown of MALAT1 attenuated HK-2 cell viability inhibition, apoptosis, and inflammation induced by HG. Then, we demonstrated that MALAT1 interacted with miR-15b-5p and miR-15b-5p targeted TLR4. MALAT1 knockdown increased miR-15b-5p levels. A miR-15b-5p inhibitor or TLR4 overexpression reversed the above effects induced by MALAT1 knockdown. Thus, our study may provide a novel therapeutic target for DN patients through MALAT1/miR-15b-5p/TLR4 signaling.

## Figures and Tables

**Figure 1:** MALAT1 and miR-15b-5p expression in DN tissues and HK-2 cells treated with NG, HM, or HG. (a) qRT-PCR analysis of MALAT1 in DN tissues. ^∗^*p* < 0.05 versus the NG group. (b) qRT-PCR analysis of MALAT1 in HK-2 cells treated with NG, HM, or HG after 12, 24, 36, or 48 h. ^∗^*p* < 0.05 versus the NG group. (c) qRT-PCR analysis of miR-15b-5p in HK-2 cells treated with NG, HM, or HG. ^∗^*p* < 0.05 versus the NG group.

**Figure 2:** Knockdown of MALAT1 attenuates HG-induced cell viability inhibition, apoptosis, and expression of inflammatory cytokines in HK-2 cells. (a) qRT-PCR analysis of MALAT1 in HK-2 cells after transfection with si-MALAT1 or si-NC. ^∗^*p* < 0.05 versus the HG or si-NC group. (b) Cell viability by CCK-8 assay. ^∗^*p* < 0.05 versus the HG or si-NC group. (c, d) Cell apoptosis by TUNEL assay. ^∗^*p* < 0.05 versus the HG or si-NC group. (e–g) ELISA analysis of TNF-*α*, IL-1*β*, and IL-6. ^∗^*p* < 0.05 versus the HG or si-NC group.

**Figure 3:** MALAT1 binds with miR-15b-5p, and an miR-15b-5p inhibitor reverses HG-induced HK-2 cell activity via MALAT1. (a) The binding sites between MALAT1 and miR-15b-5p and MALAT1-Mt sequence in the binding sites. (b, c) MALAT1 luciferase activity in HK-2 cells cotransfected with MALAT1-Wt or MALAT1-Mt vector and miR-15b-5p mimics or mimics NC. ^∗^*p* < 0.05 versus the mimics NC group. (d) Anti-Ago2 RIP was carried out in HK-2 cells; then, the amount of MALAT1 or miR-15b-5p associated with Ago2 was detected by qRT-PCR. (e) Quantification of miR-15b-5p levels by qRT-PCR analysis in HK-2 cells transfected with si-MALAT1 under NG and HG conditions. (f, g) TLR4 mRNA by qRT-PCR analysis and protein levels by western blot analysis, (h) cell viability by CCK-8 assay, (i, j) cell apoptosis by TUNEL assay, and (k) TNF-*α* levels by ELISA analysis were evaluated in HG-induced HK-2 cells cotransfected with si-MALAT1 and miR-15b-5p inhibitor. ^∗^*p* < 0.05 versus the HG+si-MALAT1 group.

**Figure 4:** miR-15b-5p negatively regulates TLR4, and MALAT1 regulates TLR4 expression via miR-15b-5p. (a) TLR4 complementary sequences of wild-type (Wt) and mutant-type (Mt) TLR4 are shown with the miR-15b-5p sequence. (b) The inhibitory effect of miR-15b-5p on TLR4 3′-UTR in HK-2 cells transfected with TLR4 3′-UTR by Luciferase reporter assay. ^∗^*p* < 0.05 versus the mimics NC group. (c) Western blot analysis of TLR4 in HG-stimulated HK-2 cells transfected with miR-15b-5p mimics or mimics NC. (d) Cell viability by CCK-8 assay, (e, f) cell apoptosis by TUNEL assay, and (g) TNF-*α* levels by ELISA analysis were examined in HG-induced HK-2 cells cotransfected with si-MALAT1 and vector TLR4. ^∗^*p* < 0.05 versus HG+si-MALAT1+vector TLR4.

**Table 1:** Clinical characteristics of DN patients.

Case number	Sex (M/F)	Age (years)	BMI (kg/m^2^)	SBP (mmHg)	DBP (mmHg)	Hb (g/L)	Scr (umol/L)	ALB (g/L)	TC (mmol/L)	Proteinuria (g/d)	HbA1c (%)	Duration of DM (years)	Retinopathy (yes/no)
1	M	41	22.1	120	80	92	112	31.9	3.56	6.17	6.84	4	Yes
2	F	53	23.4	125	85	111	106	33.4	6.92	5.29	7.04	6	Yes
3	F	53	22.3	169	90	87	69	42	3.49	3.77	10.05	6	Yes
4	M	51	22.6	179	101	107	103	44.5	2.82	1.03	6.5	5	Yes
5	F	41	26.7	169	88	74	151	26.2	6.05	5.23	8.3	7	No
6	F	51	23.6	107	65	121	106	43.9	4.05	0.51	4.43	5	No
7	M	50	24.8	148	108	128	105	26.8	6.32	6.2	10.1	4	Yes
8	M	46	27.5	153	97	110	167	23.5	7.3	10.12	5.6	7	Yes
9	F	53	25.4	130	92	127	126	39.8	6.98	2.81	6.1	8	No
10	F	47	23.5	122	84	96	77	30.1	4.59	5.93	4.87	4	Yes
11	M	42	28.9	219	137	123	119	25.8	4.48	7.59	5.4	5	Yes
12	F	45	22.8	134	99	86	88	29	6.03	4.19	5.8	6	Yes
13	F	65	27.4	146	86	101	212	19.5	12.53	11.23	6.1	8	Yes
14	F	48	24.6	130	80	97	74	35.3	5.2	2.46	11.9	6	No
15	F	56	27.4	145	73	118.8	86	40.8	9.06	2.3	9.74	5	Yes
16	F	52	25.2	120	80	97	130	38.4	4.15	4.17	7.74	7	No
17	F	50	22.7	110	70	104.4	67.1	40	4.09	0.53	9.45	5	Yes
18	M	45	23.2	142	90	78.3	259	36.2	2.58	4.995	5.7	6	Yes

Abbreviations: BMI: body mass index; SBP: systolic blood pressure; DBP: diastolic blood pressure; Hb: hemoglobin; Scr: serum creatinine; TC: total cholesterol; ALB: serum albumin.

**Table 2:** qRT-PCR primers.

Primer names	Sequences (5′-3′)	
MALAT1	Forward	GCCTGGAAGCTGAAAAACGG
	Reverse	TGGAAAACGCCTCAATCCCA
miR-15b-5p	Forward	TAGCAGCACATCATGGTTTACA
	Reverse	TGCGTGTCGTGGAGTC
*β*-Actin	Forward	GATCATTGCTCCTCCTGAGC
	Reverse	ACTCCTGCTTGCTGATCCAC
U6	Forward	GCUUCGGCAGCACAUAUACUAAAAU
	Reverse	CGCUUCACGAAUUUGCGUGUCAU

## Data Availability

The data used to support the findings of this study are included within the article.
